The article "Evaluation Model of Regional Comprehensive Disaster Reduction Capacity under Complex Environment" was published in 2022. Journal: J Environ Public Health.

# Evaluation Model of Regional Comprehensive Disaster Reduction Capacity under Complex Environment

**DOI:** 10.1155/2022/1593536

**Published:** 2022-09-05

**Authors:** Jiahu Wang, Ming Li, Ping Lin

**Affiliations:** ^1^School of Hydrology and Water Resources, Hohai University, Jiangsu, Nanjing 210098, China; ^2^Center of Hydrology and Water Resources Investigation of Sichuan Province, Chengdu 610000, China

## Abstract

In order to realize the evaluation of regional comprehensive disaster reduction capacity in a complex environment, an evaluation model of regional comprehensive disaster reduction capacity in a complex environment based on remote sensing monitoring and data image feature analysis is proposed. According to the geographical location and scale of disaster spots and the parameter analysis of the model of disaster-bearing bodies around the disaster spots, the remote sensing monitoring method is adopted to extract the geographical remote sensing images of regional disaster spots in a complex environment. The collected geographical remote sensing images of regional disaster points under the complex environmental background are filtered and preprocessed, and the texture parameters of the geographical remote sensing images of regional disaster points under the complex environmental background are recognized by combining the method of image texture feature extraction. Based on the method of tone mapping, the rapid filtering and feature analysis of the geographical remote sensing images of regional disaster points under the complex environmental background are carried out, and the time, position, damage, and so on in the geographical remote sensing images of regional disaster points under the complex environmental background are analyzed. By using the method of parameter analysis and gradient operator operation, a comparison model of geographical remote sensing images of regional disaster points under the complex environmental background is established, and the reliability evaluation of regional comprehensive disaster reduction ability under the complex environmental background is realized according to the method of contrast and detail significance enhancement. The test shows that this method has high accuracy in evaluating regional comprehensive disaster reduction capability under a complex environment, high accuracy in marking the geographical location of regional disaster points under a complex environment, and good fusion performance and reliability of regional comprehensive disaster reduction capability evaluation parameters.

## 1. Introduction

At present, most of the researches on geological disasters focus on hazard zoning and risk analysis, and most of them are static analysis, while the comprehensive loss risk analysis and dynamic assessment of geological disasters are few. However, in practice, geological disasters are uncertain and random, so it is necessary to evaluate the losses caused by geological disasters by dynamic simulation. In this study, through multisource data fusion and key mechanism research, the technical system of risk dynamic assessment of debris flow geological hazards was established, and the risk dynamic assessment of debris flow geological hazards was carried out, which deepened the research on the formation mechanism of debris flow hazards, broadened the application fields and methods of risk assessment of geological hazards, and supplemented the shortcomings and defects of the existing assessment contents [1]. It provides a new idea and method for the study of geological disaster risk in China and has certain theoretical significance. China is one of the countries with the most serious geological disasters in the world. The geological environment in the mountainous area of southeast Jilin Province is complicated, and geological disasters such as collapse, landslide, and debris flow occur frequently every year during flood season. The theoretical research on the dynamic risk assessment of debris flow geological disasters in southeast mountainous areas of Jilin Province can be directly applied to the investigation and evaluation of geological disasters, which can provide theoretical guidance and a scientific basis for the defense work in southeast mountainous areas of Jilin Province, promote the research of theoretical basis and technology of geological disaster risk analysis in Jilin Province, and improve the level of geological disaster prevention and control [2]. The application research of dynamic risk assessment of debris flow geological disasters provides a better guarantee for the monitoring and early warning system. It can provide a basis for the organization's transfer decision in advance when geological disasters occur, and it is of great significance for ensuring the safety of people's lives and property [3].

With the development of hyperspectral remote sensing monitoring image processing technology, people pay attention to the application of hyperspectral imaging technology in food comprehensive disaster reduction capability evaluation and tracking identification. In the detection of regional disaster points under a complex environment, the program model of regional disaster point geographic remote sensing image under the complex environmental background is established by combining hyperspectral technology, and the spatiotemporal distribution characteristics of disaster-causing factors in regional disaster point geographic remote sensing image under the complex environmental background are analyzed by texture distribution domain characteristics [4–6]. Using the automatic image segmentation technology, combined with the fusion of spatiotemporal distribution characteristics and texture distribution parameters of disaster-causing factors in geographical remote sensing images of regional disaster spots under the complex environmental background, the retrospective identification of comprehensive disaster reduction capability evaluation of regional disaster spots under the complex environmental background is carried out, and the accuracy and reliability of comprehensive disaster reductiaon capability evaluation of regional disaster spots under the complex environmental background are improved [7]. This paper studies the evaluation method of comprehensive disaster reduction capability of regional disaster points in a complex environment, filters the collected geographical remote sensing images of regional disaster points in a complex environment, and realizes the texture parameter identification of geographical remote sensing images of regional disaster points in a complex environment with the method of image texture feature extraction. The research on the evaluation method of comprehensive disaster reduction capability of regional disaster points in a complex environment has attracted great attention.

This paper studies the image information processing technology with the regional disaster point geographic remote sensing image processing as the core technology under the complex environmental background, combined with the image texture feature extraction and parameter analysis, to achieve the regional disaster point geographic remote sensing image parameter recognition under the complex environmental background, and finally carries out simulation test. It shows the superior performance of the proposed method in improving the ability of regional disaster spot geographic remote sensing image detection under the complex environmental background.

## 2. Evaluation Method Based on Hyperspectral Remote Sensing Monitoring Image Technology

### 2.1. Research Content

1. Based on field survey and investigation and interpretation and analysis of satellite remote sensing data, the pregnant environment, disaster-bearing body, and disaster-causing factors of debris flow disaster in the study area are determined, and the temporal and spatial distribution characteristics of rainfall of disaster-causing factors of debris flow disaster and its correlation with debris flow disaster are analyzed.
2. According to the results of the debris flow disaster system analysis and natural disaster risk index method, select the representative indicators of debris flow disaster risk assessment, calculate the weight of indicators based on the PSO-AH method, construct the debris flow disaster risk assessment index system in the study area, and make a dynamic assessment of debris flow disaster risk in the study area from 1956 to 2021.
3. According to the theory of risk management, combined with the dynamic changes of risk influencing factors of debris flow disaster and the results of risk dynamic evaluation, put forward reasonable risk prevention countermeasures and implementation ways.

### 2.2. Hyperspectral Remote Sensing Monitoring Image Acquisition

In order to realize the comprehensive disaster reduction capability evaluation of regional disaster points in a complex environment based on hyperspectral remote sensing monitoring image technology, the method of adaptive global tone mapping was used to collect regional disaster points' geographic remote sensing images in a complex environment, and combined with the edge detection method [8, 9], an automatic segmentation model of spatiotemporal distribution characteristics and texture distribution domain of regional disaster points' geographic remote sensing images in a complex environment was established. The filtering detection and analysis model of spatiotemporal distribution characteristics texture distribution domain of regional disaster point remote sensing images under the complex environmental background is constructed, and the pixels per inch sampling structure of spatiotemporal distribution characteristics texture distribution domain of regional disaster point remote sensing images under the complex environmental background is obtained [10]. The texture distribution characteristic quantity of spatiotemporal distribution characteristics texture distribution domain of regional disaster point remote sensing images under the complex environmental background is represented, and the image is collected by using a Gaussian window with a window of 5 × 5, and the expression of spatiotemporal distribution characteristics texture characteristics of regional disaster point remote sensing images under the complex environmental background is as follows:

(1) $$\begin{array}{c} I\left(x\right)=\mathrm{A\rho x}+\frac{1-\rho_{2}c_{2}/\rho_{1}c_{1}}{1+\rho_{2}c_{2}/\rho_{1}c_{1}}, \end{array}$$

where *A* is the bottom feature, *ρ* is the color contrast difference of other pixels, *x* is the feature atlas, *ρ*_1_ is the feature fusion coefficient, *c*_1_ is the feature parameter of adjacent layers, and *ρ*_2_ is the convolution operation parameter of 3 × 3. In the local area of *N* × *N*, the spatiotemporal distribution feature texture distribution domain of regional disaster point geographic remote sensing image disaster factors under the complex environmental background is segmented, and the disaster factor of regional disaster point geographic remote sensing image under the complex environmental background is obtained.

(2) $$\begin{array}{c} J\left(x\right)=\frac{2\pi^{2}f^{2}}{c^{3}\rho }\left(\frac{4}{3}\eta +\frac{r-1}{c_{p}}k\right)+A, \end{array}$$

where *f* is the frequency of the feature map in three dimensions: width and depth, *c* is the high-spectral intensity of regional disaster point quality under the complex environmental background, *η* is the regression parameter of regional disaster point geographic remote sensing image under the complex environmental background, *k* is the joint parameter, and *r* is the statistical characteristic quantity. By using the method of prediction probability density analysis of the model, the difference of degree of spatiotemporal distribution characteristic texture distribution domain of disaster factors in regional disaster point geographic remote sensing image under the complex environmental background is obtained. Using the Gaussian filtering method, the weighted analysis of the feature distribution domain is carried out, and the image acquisition model is established. The geographic remote sensing image acquisition output of regional disaster points under the complex environmental background is as follows:

(3) $$\begin{array}{c} a_{k}={\left(\sum {}_{k}+\varepsilon U\right)}^{-1}M\Delta_{s}u^{\left(n\right)}\left(x,y\right)+N\Delta_{t}, \end{array}$$

where ∑_*k*_ is a single image enhancement coefficient, *N* is a tone mapping parameter, *ε* is a high-spectral detail adjustment parameter of regional disaster point quality under the complex environmental background, *U* is a multiple of detail enhancement, and Δ_*t*_ is a smooth function. According to the edge detection result of the spatiotemporal distribution characteristic texture distribution domain of disaster factors in geographical remote sensing images of regional disaster points under the complex environmental background, combined with the template matching method, fuzzy feature detection of geographical remote sensing images of regional disaster points in the complex environmental background is carried out, and the texture detection model of spatiotemporal distribution characteristics of disaster factors in geographical remote sensing images of regional disaster points in the complex environmental background is established by Re algorithm.

### 2.3. Hyperspectral Preprocessing and Image Feature Extraction

The collected geographic remote sensing images of regional disaster points in the complex environmental background are filtered and preprocessed, and the texture parameters of the geographic remote sensing images of regional disaster points in the complex environmental background are recognized by combining the method of image texture feature extraction [11, 12]. The texture distribution domain matching model of the spatiotemporal distribution characteristics of disaster-causing factors in geographic remote sensing images of regional disaster points in the complex environmental background is established by statistical feature analysis and similarity detection [13], and the hyperspectral preprocessing is carried out by combining the matching filter detection. Using the nonlinear filter, the nonlinear filter function of texture distribution detection of the spatiotemporal distribution characteristics of disaster factors in geographical remote sensing images of regional disaster points under the complex environmental background is obtained as follows:

(4) $$\begin{array}{c} S_{m}=\frac{\left(F_{m}^{G},F_{m}^{P}\right)}{\left\|F_{m}^{G}\right\|\cdot \left\|F_{m}^{P}\right\|}, \end{array}$$

where *F*_*m*_^*G*^ is the filtered image and *F*_*m*_^*P*^ is the bilateral filtering function. According to the analysis of the relevant smooth function, the texture distribution domain of the spatiotemporal distribution characteristics of disaster-causing factors in the geographical remote sensing image of regional disaster points under the complex environmental background is divided into blocks, which are expressed as follows:

(5) $$\begin{array}{c} R_{w}={\left|\frac{r_{2}-r_{1}}{r_{2}+r_{1}}\right|}^{2}, \end{array}$$

(6) $$\begin{array}{c} y_{T}=W_{i}^{T}M_{T}, \end{array}$$

where *r*_1_ is the similarity between pixels, *r*_2_ is the correlation coefficient of brightness term, *M*_*T*_ is the halo that the image will produce, and *W*_*i*_ is the hyperspectral texture component of regional disaster point quality under the complex environmental background. After *M*_*T*_ projection, the spatiotemporal distribution characteristics and texture distribution domain of disaster causing factors are obtained. By using subspace mapping, a fusion model of spatiotemporal distribution characteristics of disaster causing factors in hyperspectral remote sensing monitoring images is constructed, and the texture distribution set is obtained as follows:

(7) $$\begin{array}{c} C=\frac{\rho \upsilon_{c}d}{\mu }\\ =\frac{\upsilon_{c}d}{\nu }, \end{array}$$

where *υ*_*c*_ is the pixel set after the global mapping of the input image, *d* is the distribution distance of pixel feature points, *ν* is the lost detail information, and *μ* is the detail compensation output. By adopting the regional template matching method, the difference of degree of the internal information of the regional disaster point geographic remote sensing image under the complex environmental background is obtained [14], and the spatiotemporal distribution characteristics of disaster-causing factors and the texture detection output of the regional disaster point geographic remote sensing image under the complex environmental background are as follows:

(8) $$\begin{array}{c} t_{Ii}=\frac{2}{{\left[4\;\cos^{2}\;kD_{i}+\left(S_{21}+S_{12}\right)\sin^{2}\;kD_{i}\right]}^{1/2}}, \end{array}$$

where *D*_*i*_ is the brightness component, *S*_12_ is the brightness order error, *S*_21_ is the hyperspectral information entropy of regional disaster point quality under the complex environmental background, and *k* is the information richness. Based on Radon scale transformation, the texture feature extraction results of spatiotemporal distribution characteristics of disaster-causing factors in geographical remote sensing images of regional disaster points under the complex environmental background are as follows:

(9) $$\begin{array}{c} t_{I}=\prod_{i=1}^{n}t_{Ii}\\ =\prod_{i=1}^{n}\frac{2}{{\left[4\;\cos^{2}\;kD_{i}+\left(S_{21}+S_{12}\right)\sin^{2}\;kD_{i}\right]}^{1/2}}, \end{array}$$

where ∏_*i*=1_^*n*^*t*_*Ii*_ means cascade summation of similarities. Based on the subjective quality evaluation method, the feature quantity of edge contour of geographical remote sensing image of regional disaster point under the complex environmental background is

(10) $$\begin{array}{c} K=\frac{I^{c}\left(y\right)}{A^{c}}\\ =\frac{2}{{\left[4\;\cos^{2}\;kD_{i}+\left(S_{21}+S_{12}\right)\sin^{2}\;kD_{i}\right]}^{1/2}}, \end{array}$$

where *D*_*i*_ is the natural image statistical model parameter and *S*_12_ and *S*_21_, respectively, represent the joint feature quantity. Therefore, the fusion model of regional disaster point geographic remote sensing images under the complex environmental background is constructed, and the fusion output of spatial and temporal distribution characteristics of disaster factors in hyperspectral remote sensing monitoring images is as follows:

(11) $$\begin{array}{c} I\left(x\right)=J\left(x\right)t\left(x\right)+A\left(1-t\left(x\right)\right), \end{array}$$

where *J*(*x*) is the order difference of the original image, *t*(*x*) is the gradient coefficient, *A* is the gain, and *I*(*x*) is the pixel set. According to the above feature extraction algorithm, according to the fusion results of regional disaster point remote sensing images in the complex environmental background, combined with the spatiotemporal distribution feature texture distribution domain of disaster-causing factors in regional disaster point remote sensing images in the complex environmental background, information is segmented, and hyperspectral preprocessing and image texture extraction are carried out [15].

## 3. Analysis of Regional Disaster Point Structure under Complex Environmental Background

### 3.1. Analysis of Spatial and Temporal Distribution Characteristics of Disaster-Causing Factors

The spatial and temporal distribution characteristics of disaster factors, dynamic distribution characteristics of disasters, and geographical characteristics of disaster points in geographical remote sensing images of regional disaster points under the complex environmental background are analyzed. Firstly, the spatial and temporal distribution characteristics of disaster factors in geographical remote sensing images of regional disaster points under the complex environmental background are analyzed. Combined with geographical remote sensing quality hyperspectral remote sensing monitoring images of disaster spots in frozen regions, the spatiotemporal distribution characteristics of disaster factors, and texture distribution domain, the edge fuzzy set of the spatiotemporal distribution characteristics of disaster factors is obtained as follows:

(12) $$\begin{array}{c} p\left(x,t\right)=\frac{2\pi^{2}f^{2}\eta }{c^{3}\rho }\left(\frac{4}{3}+\frac{r-1}{k}k^{\prime }\right), \end{array}$$

where *f* is the sampling spectrum, *k* is the dynamic distribution coefficient of the spatiotemporal distribution characteristics of disaster-causing factors, *η* is the hyperspectral spectrum separation coefficient, and *k*′ is the differential component of the dynamic distribution coefficient of the spatiotemporal distribution characteristics of disaster-causing factors. The low illumination image is enhanced, and the regional feature block detection method is adopted to construct the texture and configuration parameters of the spatiotemporal distribution characteristics of disaster-causing factors in the geographical remote sensing image of regional disaster points under the complex environmental background [16–18]. The output is as follows:

(13) $$\begin{array}{c} x_{i}\left(t\right)=I\left(x_{i},y_{i}\right)+\left[\begin{array}{cc} I_{x}\left(x_{i},y_{i}\right) & I_{y}\left(x_{i},y_{i}\right) \end{array}\right], \end{array}$$

where *I*(*x*_*i*_, *y*_*i*_) is the objective measurement enhanced image, *I*_*x*_(*x*_*i*_, *y*_*i*_) is the *X*-axis sample component of the image, and *I*_*y*_(*x*_*i*_, *y*_*i*_) is the *Y*-axis sample component of the image. By using the methods of parameter analysis and gradient operator operation, a color fusion model is established, and a fine semantic segmentation method is adopted to detect the fuzzy edge and block the geographical remote sensing image of regional disaster points under the complex environmental background, which is expressed as follows:

(14) $$\begin{array}{c} \left\{\begin{array}{c} G_{j}^{\max}==-\sigma \frac{\partial u\left(x,t\right)}{\partial x}\;\left.j\in \left\{1,\ldots ,p\right\}\right.,\\ G_{j}^{\max}=\underset{i=1,\ldots ,N}{\max}\left(G_{j}\left({\overset{⟶}{x}}_{i}\right)\right),\\ k^{\prime }=\frac{k}{\eta c_{p}},\;j\in \left\{1,\ldots ,p\right\}, \end{array}\right. \end{array}$$

where *σ* is the image color difference contrast, $G_{j}\left({\overset{⟶}{x}}_{i}\right)$ is the saturation error, *c*_*p*_ is the color difference, and *η* is the detection efficiency. According to the above analysis, combined with the texture distribution of the spatiotemporal distribution characteristics of the disaster-causing factors in the geograaphical remote sensing images of regional disaster points under the complex environmentl background, spectral analysis is adopted to detect and analyze the spatiotemporal distribution characteristics of the disaster-causing factors [19], and the spatiotemporal distribution characteristic components of the disaster-causing factors in the geographical remote sensing images of regional disaster points under the complex environmental background are extracted. Fuzzy degree detection, combined with the distribution of dynamic feature points of geographical remote sensing images of regional disaster points, and hyperspectral remote sensing monitoring images are used to match the spatial and temporal distribution characteristics of disaster-causing factors. The output is

(15) $$\begin{array}{c} \left[\begin{array}{c} x\\ y \end{array}\right]=\frac{C_{\beta }}{\text{Sin}\beta }\\ =\frac{C_{\gamma }}{\text{Sin}\gamma }, \end{array}$$

where

(16) $$\begin{array}{c} C_{\gamma }=U+\frac{\sin\;\gamma_{2}}{c_{\gamma_{2}}}+\frac{\sin\;\beta_{2}}{\beta_{2}}, \end{array}$$

where *C*_*β*_ is color contrast difference pair, *C*_*γ*_ is color contrast significance, *β* is Gaussian blur coefficient, and *γ* is joint spectrum. In order to detect the texture distribution of the spatiotemporal distribution characteristics of disaster-causing factors in geographical remote sensing images of regional disaster points under the complex environmental background, the feature analysis and detection of geographical remote sensing images of regional disaster points under the complex environmental background are realized by fusing brightness and contrast [20].

### 3.2. Analysis of Dynamic Distribution Characteristics of Disasters

According to the texture analysis results of the spatiotemporal distribution characteristics of disaster-causing factors in the geographical remote sensing images of regional disaster points in the complex environmental background [21, 22], the disaster dynamic distribution characteristics of the geographical remote sensing images of regional disaster points in the complex environmental background are analyzed, and the subpixel parallax of the geographical remote sensing images of regional disaster points in the complex environmental background is obtained as follows:

(17) $$\begin{array}{c} g\left(x,y\right)=\frac{m\;\cos\;\theta_{i}-\sqrt{n^{2}-\;\sin^{2}\theta_{i}}}{m\;\cos\;\theta_{i}+\sqrt{n^{2}-\;\sin^{2}\theta_{i}}}, \end{array}$$

where *θ*_*i*_ is the gray value of water parallax of geographical remote sensing images of regional disaster points in the complex environmental background, *n* is the significance value determined by color contrast difference, and *m* is the dynamic distribution characteristics of disasters. In the process of multistage downsampling, the detection matching values of the dynamic distribution characteristics of regional disaster points in the complex environmental background are as follows:

(18) $$\begin{array}{c} L=\beta F\left(x,y\right)+Z_{s1}\\ =\frac{\rho_{1}c_{1}}{\cos\;\theta_{i}}, \end{array}$$

where *β* is a multifeature fusion point, *F*(*x*, *y*) is a significant map detail of disaster dynamic distribution characteristics of geographical remote sensing images of regional disaster points under the complex environmental background, *Z*_*s*1_ is a threshold value of distribution of geographical remote sensing images of regional disaster points under the complex environmental background, *ρ*_1_ is a European cluster of distribution of water-bearing characteristic points of geographical remote sensing images of regional disaster points under the complex environmental background, *c*_1_ is a joint evaluation coefficient, *θ*_*i*_ is a horizontal offset, *m*_*l*_ is the weak texture set of the spatial and temporal distribution characteristics of disaster-causing factors in the geographical remote sensing images of regional disaster points under the complex environmental background [23, 24], and *δ*_*l*_^2^ is the interval of water-bearing points distribution in the geographical remote sensing images of regional disaster points under the complex environmental background.

### 3.3. Analysis of Geographical Characteristics of Disaster Points

The geographical characteristics of disaster points mainly investigate and verify the geographical location and scale of disaster points, investigate the disaster-bearing body around the disaster points and the relevant socio-economic data of the region, and verify whether the land use type interpreted by remote sensing is accurate, so as to provide a reference for the selection of key indicators for the dynamic assessment of geological disaster risk induced by extreme precipitation in mountain areas and provide the basis for the verification of the results of the dynamic assessment of geological disaster risk induced by extreme precipitation in mountain areas [25]. The characteristics of geographical remote sensing images of regional disaster points under the complex environmental background are analyzed, and the rainfall characteristics of inducing factors are detected. The spectral wavelength coefficient is as follows:

(19) $$\begin{array}{c} L=J\left(w,e\right)-\sum_{i=1}^{N}a\left[4\;\cos^{2}\;kD_{i}+\left(S_{21}+S_{12}\right)\sin^{2}\;kD_{i}\right], \end{array}$$

where *J*(*w*, *e*) is the initial wavelength, *a* is the geographical remote sensing spatial characteristic quantity of regional disaster points under the complex environmental background, and *D*_*i*_ is the remote sensing spectral reflection coefficient. The reflection coefficient of regional disaster point quality hyperspectral disaster regionality under the complex environmental background is defined, and the grayscale increase part is obtained as follows:

(20) $$\begin{array}{c} \text{Dark}\left(x\right)=p_{a}e^{j\left(wt-k\cdot r\right)}+\underset{c\in \left\{r,g,b\right\}}{\min}R, \end{array}$$

where *p*_*a*_ is the Lab spatial feature after Gaussian smoothing, *e*^*j*(*wt* − **k** · **r**)^ is the gray rate of regional disaster points under the complex environmental background, and *R* is the scale. Combined with convolution scale analysis, the rainfall characteristics of regional disaster point remote sensing images in a complex environment are detected [26]. Combined with the spatial and temporal distribution characteristics of disaster-causing factors and texture analysis results, a comparison model of regional disaster point remote sensing images in a complex environment is established. According to the method of contrast and detail significance enhancement, the reliability detection of regional disaster point quality in a complex environment is realized.

## 4. Experimental Analysis

### 4.1. Experimental Preparation

The simulation experiment of comprehensive disaster reduction capability evaluation of regional disaster sites in a complex environment is based on MATLAB simulation software and SPECIM Spectral Camera hyperspectral analysis, and the remote sensing image data includes “Gaofen-1” satellite image data. It includes four types of data, including 2-meter panchromatic, 8-meter multispectral, fusion of both, and 16-meter multispectral, which are all from the geographic and national monitoring cloud platform. The DEM data used in this study comes from DLR-DEM data, one of the SRTM data provided by Deutsche Zentrum Firluft-und Raum Fahrt, with an elevation accuracy of 6–16 m.

The meteorological data comes from China Meteorological Science Data Network (https:/lcdc.nmic.cn/). According to the continuity and the longest period standard of meteorological data of each station, the daily meteorological data of all meteorological stations around the study area from 1956 to 2021 are selected. MSRA10K data set and THUR15K data set are used as test sets, and 200 figures were selected from the two datasets as training parameters. The detected regional disaster point samples under the complex environmental background were divided into 15 groups. The basic geographic data and ecological environment data such as the detailed administrative boundary and topographic contour of a county are from the geological environment department of the Department of land and resources of a province; the geological and geomorphological data are from the data provided by the geological environment department of the Department of land and resources of a province; the land use data comes from the data provided by the geographic situation monitoring cloud platform; the soil type data is from the national soil type digital map provided by the geographic situation monitoring cloud platform; the hydrogeological data comes from the geological science data sharing network of the Chinese Academy of Geological Sciences. The field investigation scene of the staff is shown in Figure 1.

In the part of data processing, in the process of digitizing geological maps, identifying and extracting disaster points, and identifying risk factors of geological disasters, some indicators need to be obtained by remote sensing interpretation technology. In order to meet the requirements of the project, the project team adopted aerial images (scale 1:10,000, resolution 0.5 m, Tonghua County) and DLR-DEM digital elevation data as the basic maps for digitizing geological disasters. The related data processing mainly includes digitization of geological topographic maps, extraction of geological factors, and remote sensing interpretation of land use types. Geological factors are mainly extracted and analyzed by Spatial AnalysisTools in ArcToolBox Toolbox in ArcGIS10.2, including related factors such as slope and aspect. The extraction methods are as follows.

Slope indicates the degree of inclination of a point on the ground surface relative to the horizontal plane, and aspect is a quantifier to describe the inclination of that point. The value of the slope of a point on the surface is the angle between the tangent plane of the surface and the horizontal plane, and the slope direction of the point is the azimuth angle projected on the horizontal plane by the tangent plane along the maximum inclination direction vector. In this research, ArcGIS10.2 software is used to generate data on slope and aspect.

The experimental images and data are from Microsoft Azure Data Markets Free Datasets, which provide free data sets covering everything from agriculture to weather, and the collected geographical remote sensing images of regional disaster points under the complex environmental background are filtered and preprocessed, and the collected original hyperspectral remote sensing monitoring images are obtained as shown in Figure 2.

### 4.2. Experimental Results and Analysis

According to the sampling results of the above-mentioned experimental samples, the comprehensive disaster reduction capability of regional disaster spots under the complex environmental background is evaluated. The spatial and temporal distribution characteristics of disaster-causing factors, the dynamic distribution characteristics of disasters, and the rainfall characteristics of inducing factors in the geographical remote sensing images of regional disaster spots under the complex environmental background are analyzed by using the hyperspectral remote sensing monitoring image analysis method, and the results of disaster risk evaluation and comprehensive disaster reduction feature extraction are shown in Figure 3.

According to the analysis of Figure 3, this method can effectively extract the quality correlation characteristics of regional disaster points under the complex environmental background, and the performance curve of comprehensive disaster reduction capability evaluation is shown in Figure 4.

According to the analysis of Figure 4, the accuracy of the regional comprehensive disaster reduction ability evaluation by using this method in the complex environmental background is high; the geographical location of regional disaster points in the complex environmental background is accurate; and the parameter fusion performance of regional comprehensive disaster reduction ability evaluation is good, and the reliability is high. Combined with the evaluation results of disaster risk reduction ability in this study, the different villages and towns in the study area show obvious differences in disaster risk reduction ability, which is determined by the social and economic conditions of each region. In the towns around an urban area, the ability of disaster prevention and mitigation against debris flow disasters has been significantly strengthened with the development of time, which is mainly reflected in the increasingly perfect establishment of disaster emergency agencies and the establishment of disaster monitoring sites from scratch. In the early stage, due to the lack of disaster-related emergency facilities, there was no effective emergency plan when disasters came, which caused a lot of losses. Because of this, these areas also continuously strengthened the publicity and construction at the level of residents' disaster cognition, but there were also shortcomings. Through the investigation, it is found that the disaster emergency plan is still not perfect, the real-time monitoring technology before the disaster, and the social and economic repair measures after the disaster are still relatively lacking, which causes the lag in disaster prevention and control and the failure to respond in time and deal with the damage caused by the disaster reasonably. For the remote towns in the study area, there are no perfect emergency plans and institutions, and local residents still have little understanding of mudslide disasters, which is not conducive to rescue work when disasters come, resulting in a significant increase in disaster losses. Therefore, it is suggested that towns with relatively perfect social economies should establish a perfect preplan from predisaster prediction to postdisaster loss reconstruction and risk sharing as soon as possible. In remote areas, it is urgent to establish disaster monitoring sites and emergency response agencies in high-risk areas, so as to make timely responses when disasters occur. At the same time, the education and publicity about debris flow and geological disasters should be strengthened to improve residents' cognitive level, improve their ability to resist disasters, and reduce casualties and property losses.

## 5. Conclusions

Debris flow is sudden and destructive. If there are adequate emergency plans, disaster prevention measures, and early warning and evaluation systems, the postdisaster emergency rescue capability of disaster-bearing areas will be greatly improved so that the safety of the population and economy can be protected in time, and the disaster emergency system can be quickly responded to. The postdisaster reconstruction, economic recovery, disease prevention, and disaster prevention work also need effective records. The faster the recovery from the postdisaster, the more losses and negative impacts caused by the disaster will be reduced.

In this paper, the automatic image segmentation technology is adopted, and the texture distribution parameters of disaster-causing factors in geographical remote sensing images of regional disaster points under a complex environment are fused, so as to carry out retrospective identification of comprehensive disaster reduction capability evaluation of regional disaster points under a complex environment and improve the accuracy and reliability of comprehensive disaster reduction capability evaluation of regional disaster points under a complex environment. In this paper, the quality reliability detection is realized by hyperspectral detection of quality-related parameters of regional disaster points under a complex environment, such as gloss, disaster dynamic distribution characteristics, rainfall characteristics of inducing factors, and so on. The test shows that this method is more accurate and reliable in evaluating the comprehensive disaster reduction ability of regional disaster points under the complex environmental background. According to the research, the main conclusions are as follows:

1. According to remote sensing identification and statistical analysis of historical disaster data, the main geological disaster in the study area is debris flow. Its disaster points are distributed in a large number and range, and the scale of disasters is mainly small. The main hazards are farmland, roads, and houses, sometimes causing casualties.
2. In the systematic analysis of debris flow disasters in the study area, the main factors affecting debris flow disasters in the pregnant environment are stratum lithology, geological structure, topography, meteorology and hydrology, vegetation conditions, and so on. The main disaster-bearing bodies in the area are population and economic property, and the disaster-inducing factor is the flood formed by rainfall entering the surface valleys, so there is a significant positive correlation between debris flow disaster and rainfall.
3. Fully consider various factors that may affect the formation of debris flow disasters, comprehensively analyze and study the formation mechanism of regional debris flow geological disasters, and pertinently construct a comprehensive evaluation index system framework of debris flow disaster risk in localized research areas.
4. Based on the formation mechanism of natural disasters, combined with disaster-causing factors, the coupling of disaster-bearing body and disaster-bearing environment comprehensively evaluate the risk of geological disasters and the possible losses.

The next step of research can consider the following: if the rescue channel is cut off in the event of a heavy rain disaster, the loss will increase exponentially. Therefore, the local government needs to prepare emergency materials in advance, and also strengthen the protection of road traffic, respond in time, and to increase the ability to carry out rescue work; in this process, the main focus is to improve emergency facilities and ensure the transportation network, which can be studied in depth in the future.

## Figures and Tables

**Figure 1:** Field investigation scene of staff: (a) scenario 1 and (b) scenario 2.

**Figure 2:** Original hyperspectral remote sensing monitoring image: (a) binary diagram and (b) hyperspectral map.

**Figure 3:** Extraction results of spatial map distribution of disaster risk assessment and comprehensive disaster reduction: (a) risk assessment of debris flow disaster induced by extreme rainfall in mountainous areas and (b) spatial map distribution of comprehensive disaster reduction.

**Figure 4:** Performance curve of comprehensive disaster reduction capability evaluation.

## Data Availability

The raw data supporting the conclusions of this article will be made available by the authors, without undue reservation.

## References

[1] Ceola S., Domeneghetti A., Schumann G. J. P. (2022). Unraveling long-term flood risk dynamics across the murray-darling basin using a large-scale hydraulic model and satellite data. *Frontiers in Water*.

[2] Lechowska Ewa (2021). Approaches in research on flood risk perception and their importance in flood risk management: a review. *Natural Hazards*.

[3] Zuzelo P. R. (2022). Flood Risk Assessment:An Important Component of Holistic Home Safety Assessment. *Holistic Nursing Practice*.

[4] Yang R., Wu S., Gao X. (2021). An accuracy-improved flood risk and ecological risk assessment in an interconnected river–lake system based on a copula-coupled hydrodynamic risk assessment model. *Journal of Hydrology*.

[5] Chen J., uang G., Chen W. (2021). Towards better flood risk management: Assessing flood risk and investigating the potential mechanism based on machine learning models. *Journal of Environmental Management*.

[6] Yin Q., Ntim-Amo G., Ran R. (2021). Flood Disaster Risk Perception and Urban Households’ Flood Disaster Preparedness: The Case of Accra Metropolis in Ghana. *Water*.

[7] Howe Nick P., Shamini B. (2021). Flood risk rises as people surge into vulnerable regions. *Nature*.

[8] Zhao X.-e., PAN X., Wei-hong Y. (2020). Research on grassland forage hyperspectral image recognition based on variance selection and Gaussian Naive Bayes. *Journal of Optoelectronics·Laser*.

[9] Ning Y., Cui W., Zhang Z. (2020). Soil salinity inversion at different depths using improved spectral index with UAV multispectral remote sensing. *Transactions of the Chinese Society of Agricultural Engineering*.

[10] Rufat S., Botzen W. W. (2022). Drivers and dimensions of flood risk perceptions: Revealing an implicit selection bias and lessons for communication policies. *Global Environmental Change*.

[11] Jang J. H., Chang T.-H. (2022). Flood risk estimation under the compound influence of rainfall and tide. *Journal of Hydrology*.

[12] Yu Y., Yang Y., Lan L. (2020). Image style transfer network based on texture feature analysis. *Journal of Computer Applications*.

[13] Huang W., Hashimoto S., Yoshida T., Saito O., Taki K. (2021). A nature-based approach to mitigate flood risk and improve ecosystem services in Shiga, Japan. *Ecosystem Services*.

[14] Pham B. T., Luu C., Dao DV. (2021). Flood risk assessment using deep learning integrated with multi-criteria decision analysis. *Knowledge-Based Systems*.

[15] Li M., Liu C., Zhang Y. (2020). A Deep learning and intelligent recognition method of Image data for rock mineral and its implementation. *Geotectonica et Metallogenia*.

[16] Xiang C., Xu J., Wang M. (2020). Analysis of meteorological disaster factors of “planting rice in one season and crayfish in three seasons” model in hongze lake area. *Journal of Aquaculture*.

[17] Zheng J., Tao P., Dong X. (2020). Evolution characteristics of meteorological drought and assessment of risk of disaster factors in the three gorges reservoir Area. *Research of Soil and Water Conservation*.

[18] Jiao L., Wang L., Zhang Q. (2020). Temporal and spatial characteristics of hail and its impact evaluation on fruit farming in Hebei Province. *Agricultural Research In The Arid Areas*.

[19] Tang J., Li Y., Cui S. (2021). Analyzing the spatiotemporal dynamics of flood risk and its driving factors in a coastal watershed of southeastern China. *Ecological Indicators*.

[20] Wang H., Zhou J., Tang Y., Liu Z., Kang A., Chen B. (2021). Flood economic assessment of structural measure based on integrated flood risk management: A case study in Beijing. *Journal of Environmental Management*.

[21] Iizuka A. (2020). Developing capacity for disaster risk reduction: l. *Progress in Disaster Science*.

[22] Choo M., Yoon D. K. (2022). Examining the effects of the local communities’ social capital on disaster response capacity in Seoul, South Korea. *International Journal of Disaster Risk Reduction*.

[23] Pescaroli G., Velazquez O., Alcántara-Ayala I., Galasso C., Kostkova P., Alexander D. (2020). A lsbmbocordr. *International Journal of Disaster Risk Science*.

[24] Mutiarni Y. S., Nakamura H., Bhattacharya Y. (2022). The resilient community: strengthening people-centered disaster risk reduction in the merapi volcano community, java, indonesia. *Sustainability*.

[25] Sumantri S. H., Kurniadi A., Marnani C. (2021). The improvement of community capacity in facing of the landslide in sukajaya subdistrict of bogor regency. *Technium Social Sciences Journal*.

[26] Sutarja I. N., Ardana M., Gustave S. P. (2022). Disaster risk reduction of mount agung cold lava flood at the bkr. *IOP Conference Series: Earth and Environmental Science*.

